This article has been retracted.

# Protective Mechanism of Trimetazidine in Myocardial Cells in Myocardial Infarction Rats through ERK Signaling Pathway

**DOI:** 10.1155/2021/9924549

**Published:** 2021-10-05

**Authors:** Zhenjun Wu, Lihua Yu, Xinyue Li, Xuewen Li

**Affiliations:** ^1^Cardiology Department, Tianjin Huaxing Hospital, Tianjin 300270, China; ^2^Beijing Chaoyang Integrative Medicine Emergency Medical Center, Beijing 100020, China; ^3^Cardiology Department, Xianshuigu Hospital of Jinnan District, Tianjin 300350, China; ^4^Cadre's Ward, Characteristic Medical Center of Chinese People's Armed Police Force, Tijian 300350, China

## Abstract

**Objective:**

To study the protective effect of trimetazidine on myocardial cells in rats with myocardial infarction and explore its effect on ERK signaling pathway.

**Methods:**

40 SD rats were randomly divided into the sham operation group, model group, low-dose group, and high-dose group (intra-abdominal injection of trimetazidine 5 mg/kg and 10 mg/kg, respectively), construction of rat myocardial infarction model by coronary artery left anterior descending artery ligation. 7 days after surgery, the survival rate and cardiac function of each group of rats were recorded. The myocardial infarct size was detected by TTC staining. The apoptosis level of rat cardiomyocytes was detected by TUNEL staining. The content of ROS in rat cardiomyocytes was detected by DCFH-DA. Western-blot was used to detection of Caspase-3, Bcl-2/Bax, and ERK signaling pathway-related proteins in myocardial tissue.

**Results:**

Compared with the model group, the survival rate of the rats in the low-dose group and the high-dose group was significantly increased (*P* < 0.01), the cardiac function was significantly improved (*P* < 0.01), the myocardial infarct size was significantly decreased (*P* < 0.01), the level of apoptosis was significantly decreased (*P* < 0.01), the content of ROS in cardiomyocytes was significantly decreased (*P* < 0.01), the protein expression of Caspase-3 and NF-*κ*B in cardiomyocytes was significantly decreased (*P* < 0.01), and the expression of Bcl-2/Bax and p-ERK were significantly increased (*P* < 0.01).

**Conclusion:**

Trimetazidine can activate ERK signaling pathway in cardiomyocytes of rats with myocardial infarction, increase the expression of p-ERK, decrease the content of ROS in cardiomyocytes, decrease the expression of apoptotic proteins, reduce myocardial infarct size, improve cardiac function, and increase myocardial function.

## 1. Introduction

The pathogenesis of myocardial infarction (MI) is the damage or death of myocardial cells due to acute ischemia and hypoxia in coronary artery, and the patients often suffer from severe substernal or precordial crushing pain, exacerbated angina, and arrhythmia. There are approximately 3 million deaths of cardiovascular disease every year, showing an increasing trend year by year [1, 2]. Wang et al. [3] studied and found that myocardial apoptosis occurs in the MI region and infarction border region, which is controlled by a series of programs, and it can be reduced via intervention. The prompt surgical intervention and thrombolytic drugs can restore cardiac blood supply, inhibit ischemic myocardial cell death and ventricular remodeling, and significantly improve cardiac function [4]. Trimetazidine, a 3-ketoacyl-CoA thiolase inhibitor, can inhibit the oxidative phosphorylation of fat and glucose, enhance the myocardial function, and protect the myocardial cells, which is used clinically in the antiangina treatment [5]. There is research evidence that trimetazidine can reduce vascular resistance, increase coronary blood flow, obviously improve clinical symptoms of patients with coronary heart disease, and ameliorate the prognosis of MI patients [6]. Zhao et al. [7] found that trimetazidine postconditioning has a protective effect on myocardial cells after myocardial ischemia-reperfusion injury. As a kind of mitogenic signal transduction-related protein, the extracellular signal-regulated kinase (ERK) signaling pathway is involved in regulating the proliferation and survival of a variety of cells, which can directly or indirectly affect the histocyte apoptosis [8]. According to the study of Liu et al. [9], activating the ERK signaling pathway can suppress the activation of downstream ELK and nuclear factor-*κ*B (NF-*κ*B), exerting an important protective effect against myocardial injury. Currently, there are few studies on the effects of trimetazidine on the ERK signaling pathway and myocardial apoptosis in MI. In this study, therefore, the rat model of MI was established, the protective effect of trimetazidine on myocardial cells in MI rats was studied, and its possible mechanism of action was further clarified.

## 2. Materials and Methods

### 2.1. Laboratory Animals and Grouping

A total of 40 specific pathogen-free (SPF) male Sprague-Dawley rats weighing 250-300 g were purchased from the Laboratory Animal Center of Guangzhou University of Chinese Medicine, and they were adaptively fed in the SPF environment for 7 d under the humidity of (45 ± 5)%, temperature of (20 ± 2)°C and regular circadian rhythm and had free access to food and water. Before modeling, the rats were fasted for food for 12 h and randomly divided into sham group (*n* = 10), model group (*n* = 10), low-dose group (*n* = 10), and high-dose group (*n* = 10). In the model group, low-dose group, and high-dose group, the rat model of MI was established via ligation of the left anterior descending coronary artery. In the sham group, the operation was the same as that in the model group without ligating the left anterior descending coronary artery. Trimetazidine (Sigma, USA) was injected intraperitoneally in the low-dose group (10 mg/kg) and high-dose group (20 mg/kg) at 30 min before operation. An equal amount of normal saline was injected intraperitoneally in the sham group and model group.

The experimental scheme was reviewed and approved by the Laboratory Animal Ethics Committee, and all experimental operations were performed in accordance with the Guide for the Use of Laboratory Animals of the National Institutes of Health.

### 2.2. Establishment of MI Model

After anesthesia via intraperitoneal injection of pentobarbital sodium (30 mg/kg), the rats were fixed in a supine position; the hair on the neck, chest, and limbs was shaved off; and the limbs were connected to the electrocardiograph, following by disinfection and draping. The neck skin was cut using surgical scissors, the muscles were bluntly separated, and the trachea was exposed and connected to the small animal ventilator (Chengdu Techman). The thoracic cavity was cut open between the left 3^rd^ and 4^th^ intercostal space, and the heart was exposed. Then, the myocardium was punctured using the 6-0 silk thread along the left coronary artery 1 mm below the left auricle to ligate the coronary artery. The weakness in cardiac impulse, whitening of myocardium, and cyanosis of myocardial tissues accompanied with ST-segment elevation indicated the successful occlusion of the anterior descending coronary artery. Then, the chest was sutured. Within 12 h after operation, penicillin was injected intramuscularly for anti-infective treatment, and the 7-d survival rate of rats was recorded.

### 2.3. Detection of Cardiac Function

Before the end of the experiment, the cardiac function of rats was determined via M-mode echocardiography using the small animal ultrasound instrument (VisualSonics, Canada). The left ventricular ejection fraction (LVEF%), left ventricular fractional shortening (LVFS%), left ventricular internal diameter at end-diastole (LVIDd), and left ventricular internal diameter at end-systole (LVIDs) were detected using the BL-420E+ biological signal acquisition and analysis device.

### 2.4. Determination of MI Area

After the experiment, the rats were sacrificed immediately, the heart was taken, and the left ventricle was separated and weighed. After the blood was washed away with precooled normal saline, the heart tissues were sliced into about 2 mm-thick sections, added with freshly-prepared pre-heated 1% TTC solution (Sigma, USA), and incubated for 15 min in the dark, during which the mixture should be shaken intermittently for thorough staining. After that, the infarction region showed the grey white color, while the noninfarction region showed the dark red color. The sections were fixed with 4% paraformaldehyde for 30 min and photographed. Then, the MI area was calculated using the Image Pro-Plus image analysis software: MI area (%) = myocardial weight in the infarction region/myocardial weight in the ischemic region × 100%.

### 2.5. Determination of Myocardial Apoptosis

After the experiment, the rats were sacrificed immediately, the heart was taken, and the left ventricle was separated. The apoptosis of myocardial cells in the ischemic region in each group was detected using the terminal deoxynucleotidyl transferase-mediated dUTP nick end labeling (TUNEL) staining kit (Beyotime Biotechnology) strictly according to the instructions. The sections were observed and photographed under a fluorescence microscope. TUNEL-positive cells were apoptotic cells displaying yellow-green fluorescence, while TUNEL-negative cells were normal cells without fluorescence. The apoptosis level of myocardial cells in each group was calculated.

### 2.6. Determination of Level of Reactive Oxygen Species (ROS) in Myocardial Cells

The level of ROS in myocardial cells was determined using the DCFH-DA assay strictly according to the instructions of kit (Beyotime Biotechnology): after the experiment, the rats were sacrificed immediately, the heart was taken, and the left ventricle was separated. Then, the tissues were homogenized with an appropriate amount of normal saline and centrifuged at 10,000 g and 4°C for 15 min. An appropriate amount of supernatant was taken, added with 10 *μ*M of DCFH-DA, incubated at 37°C for 20 min in the dark, and washed with PBS and washing solution, followed by photography under a laser confocal microscope. Finally, the content of ROS in myocardial cells was calculated.

### 2.7. Detection of Related Protein Expressions Using Western Blotting

After the experiment, the rats were sacrificed immediately, the heart was taken, and the left ventricle was separated. After an appropriate amount of RIPA lysis buffer, 1% phosphatase inhibitor and 1% protease inhibitor were added, and the tissues were smashed using the ultrasound homogenizer and centrifuged at 12,000 rpm and 4°C for 10 min. The supernatant was taken as the total protein, and its concentration was determined. After inactivation via boiling, the protein was subjected to electrophoresis and transferred onto a PVDF membrane. Then, the target band was cut according to the molecular weight of protein, sealed with freshly-prepared 5% skim milk powder for 2 h, and incubated with the B-cell lymphoma 2 (Bcl-2), Bcl-2-associated X protein (Bax), cleaved Caspase-3, phosphorylated ERK (p-ERK), ERK, NF-*κ*B, and GAPDH antibodies (1 : 1000, Cell Signaling Technology, USA) at 4°C overnight. After the band was washed with TBST for 3 times, it was incubated again with the HRP-labeled goat anti-rabbit secondary antibodies (1 : 5000, Boster Biological Technology Co., Ltd.) at room temperature for 1 h and washed again with TBST for 3 times. Then, the mixed ECL solution was added for image development and exposure. After scanning, the protein expression level in each group was analyzed using the ImageJ software.

### 2.8. Statistical Analysis

The data in this study were expressed as mean ± standard deviation. The SPSS22.0 software (SPSS Inc., Chicago, IL, USA) was used for the data processing. Analysis of variance was performed for the comparison among groups. Welch's method was adopted in the case of heterogeneity of variance, while Bonferroni's method for pairwise comparison in the case of homogeneity of variance. *P* < 0.05 suggested that the difference was statistically significant.

## 3. Results

### 3.1. Trimetazidine Increased Survival Rate of MI Rats

The survival rate of rats in each group was recorded 7 days after modeling. The results are shown in Table 1. Compared with the sham operation group, the survival rate of the model group was significantly reduced (*P* < 0.01). Compared with the model group, the survival rate of the low-dose group and the high-dose group was significantly increased (*P* < 0.01), and there was no significant difference in the survival rate of the low-dose group and the high-dose group (*P* > 0.05). Pretreatment with trimetazidine can significantly increase the survival rate of rats with myocardial infarction (*P* < 0.05).

### 3.2. Trimetazidine Improved Cardiac Function of MI Rats

The heart function of the rats was recorded 7 days after the model was established. The results are shown in Figure 1. The LVEF%, LVFS%, LVIDd, and LVIDs of the model group were significantly lower than those of the sham operation group (*P* < 0.01). The LVEF%, LVFS%, LVIDd, and LVIDs of the low-dose group and the high-dose group were significantly higher than those of the model group (*P* < 0.01 or *P* < 0.05). LVEF%, LVFS%, LVIDd, and LVIDs in the high-dose group were significantly higher than those in the low-dose group (*P* < 0.01).

### 3.3. Trimetazidine Reduced MI Area in Rats

The MI area was determined using TTC staining at 7 d after modeling. As shown in Figure 2, compared with the sham operation group, the area of myocardial infarction in rats with myocardial infarction increased significantly (*P* < 0.01), and the area of myocardial infarction in rats in the low-dose and high-dose groups was significantly lower than in the model group (*P* < 0.01). The area of myocardial infarction in the high-dose group was significantly lower than that of the low-dose group (*P* < 0.01).

### 3.4. Trimetazidine Reduced Myocardial Apoptosis in MI Rats

The rats in each group were sacrificed at 7 d after modeling, and the number of apoptotic myocardial cells was measured using TUNEL staining. As shown in Figure 3, the number of apoptotic myocardial cells was evidently larger in the model group than that in the sham group (*P* < 0.01), while it was evidently smaller in the low-dose group and high-dose group than that in the model group (*P* < 0.01). The number of cardiomyocyte apoptosis in the high-dose group was significantly lower than that of the low-dose group (*P* < 0.01).

### 3.5. Trimetazidine Reduced ROS Content in Myocardial Cells in MI Rats

After 7 days of modeling, the rats in each group were sacrificed, and the ROS content of rat myocardial cells was detected. The results are shown in Figure 4. Compared with the sham operation group, the ROS content of myocardial infarction rats increased significantly (*P* < 0.01), the content of ROS in cardiomyocytes of rats in the low-dose and high-dose groups was significantly reduced (*P* < 0.01), and the content of ROS in the cardiomyocytes of rats in the high-dose group was significantly lower than that in the low-dose group (*P* < 0.01).

### 3.6. Trimetazidine Lowered Expressions of Apoptosis-Related Proteins in Myocardial Cells in MI Rats

Rats in each group were sacrificed 7 days after modeling, and the expression of apoptosis-related proteins in cardiomyocytes was detected. The results are shown in Figure 5. Compared with the sham operation group, the expression level of Caspase-3 in myocardial cells of rats with myocardial infarction increased significantly (*P* < 0.01), and Bcl-2/Bax decreased significantly (*P* < 0.01). The expression level of Caspase-3 in the cardiomyocytes of the low-dose and high-dose groups was significantly lower than that of the model group (*P* < 0.01), and Bcl-2/Bax was significantly higher than that of the model group (*P* < 0.01). The expression level of Caspase-3 in rat cardiomyocytes in the high-dose group was significantly lower than that in the low-dose group, and Bcl-2/Bax was significantly higher than that in the low-dose group (*P* < 0.01).

### 3.7. Trimetazidine Activated ERK Signaling Pathway in Myocardial Cells in MI Rats

The rats in each group were sacrificed at 7 d after modeling, and the expressions of ERK pathway-related proteins in myocardial cells were measured. It was found that the expression of p-ERK obviously declined in myocardial cells (*P* < 0.01) and the expression of NF-*κ*B obviously rose in the model group compared with those in the sham group (*P* < 0.01). The expression of p-ERK was significantly higher (*P* < 0.01), and the expression of NF-*κ*B was significantly lower in the low-dose group and high-dose group than those in the model group (*P* < 0.01). The expression of p-ERK in the high-dose group was significantly higher than that of the low-dose group, and the expression of NF-*κ*B was significantly lower than that of the low-dose group (*P* < 0.01) (Figure 6).

## 4. Discussion

Acute MI is an ischemic heart disease that causes necrosis or apoptosis of myocardial cells due to persistent ischemia and hypoxia of heart tissues and also a common cardiovascular disease seriously threatening human health [10]. Ischemia and hypoxia lead to a massive release of oxygen free radicals in myocardial cells, activate leukocytes to secrete a large number of inflammatory factors, produce apoptosis-related proteins, and damage cell membranes and mitochondrial membranes, thus damaging myocardial cells [11]. In this study, the rat model of MI was established, and it was found that ligating the left anterior descending coronary artery could result in myocardial ischemia and hypoxia, and obvious infarction of myocardial tissues, and significantly weaken the cardiac function of rats. Li et al. [12] found that reducing the content of oxygen free radicals in cells and protecting the mitochondrial function can effectively enhance the tolerance of cells to hypoxia and reduce the release of inflammatory factors. In this study, trimetazidine preconditioning could remarkably reduce the ROS content in myocardial cells and the MI area in MI rats in a dose-dependent manner. Under hypoxic conditions, the intracellular glycolytic pathway becomes the only way of energy supply, which can lead to massive accumulation of lactic acid, hydrogen ions, and oxygen free radicals and cause cell acidosis, thereby resulting in apoptosis. Regulating the intracellular energy metabolism pathway can effectively reduce the production of oxygen free radicals and hydrogen ions, thus protecting cells [13]. In the study of Bingham and Platt [14], it was confirmed that after ligation of the coronary artery in rats, the synthesis of high-sensitivity troponin T is greatly increased, the myocardial cell membrane is damaged, and myocardial cells are impaired. Besides, Yang et al. [15] found that trimetazidine, through inhibiting the activity of fatty acid *β*-oxidation pathway 3-ketoacyl-CoA thiolase, can raise the proportion of energy produced by aerobic oxidation of intracellular glucose, reduce the aggregation of calcium and hydrogen ions in cells, stabilize the myocardial cell membrane, and protect the myocardial cells.

As one of the classic MAPK signaling pathways, the ERK signaling pathway plays a crucial role in the proliferation and differentiation of myocardial cells, and its abnormalities can lead to cardiovascular diseases, such as coronary atherosclerosis, MI, and myocardial hypertrophy [16, 17]. The stress inside and outside myocardial cells can affect the activation of the ERK signaling pathway, and activating the ERK signaling pathway can significantly raise the phosphorylation level of ERK protein, thereby affecting the expression of the downstream target protein NF-*κ*B and regulating the cell proliferation and apoptosis [18, 19]. In this study, it was found that in myocardial cells of MI rats, the expression level of p-ERK evidently declined, while that of NF-*κ*B and apoptotic protein Caspase-3 evidently rose. After trimetazidine preconditioning, the expression of p-ERK in myocardial cells was significantly increased, the expressions of NF-*κ*B and Caspase-3in myocardial cells were decreased, and the myocardial apoptosis was weakened in MI rats. According to the study of Yao et al. [20], activating the ERK signaling pathway can regulate the proliferation and migration of endothelial cells and promote the myocardial angiogenesis. At the same time, VEGF is an activator of the ERK signaling pathway. In this study, the effect of trimetazidine on angiogenesis was not explored deeply, which, however, may also be one of the mechanisms of the protective effect of trimetazidine on myocardial cells in MI rats, and the emphasis in subsequent research.

In conclusion, this study demonstrates that trimetazidine can activate the ERK signaling pathway in myocardial cells, reduce the content of ROS in myocardial cells, lower the level of myocardial apoptosis, protect the myocardial cells, and improve the cardiac function of MI rats.

## Figures and Tables

**Figure 1:** Cardiac function of rats in each group. (a) LVEF%. (b) LVFS%. (c) LVIDd. (d) LVIDs. LVEF%, LVFS%, LVIDd, and LVIDs are obviously raised in the model group compared with those in the sham group, while the low-dose group and high-dose group have notably higher LVEF% and LVFS% and larger LVIDd and LVIDs than model group. ^∗∗^*P* < 0.01 vs. model group, ^##^*P* < 0.01 vs. sham group.

**Figure 2:** Measurement of MI area. (a) TTC staining. (b) statistical diagram of MI area. The MI area in rats is evidently increased in the model group compared with that in the sham group, while it is evidently decreased in the low-dose group and high-dose group compared with that in the model group. .^∗∗^*P* < 0.01 vs. model group, ^##^*P* < 0.01 vs. sham group.

**Figure 3:** Number of apoptotic myocardial cells detected via TUNEL staining. (a) TUNEL staining. (b) Statistical diagram of TUNEL-positive cells (scale bar = 50 *μ*m). The number of apoptotic myocardial cells is evidently larger in the model group than that in the sham group, while it is evidently smaller in the low-dose group and high-dose group than that in the model group. ^∗∗^*P* < 0.01 vs. model group, ^##^*P* < 0.01 vs. sham group.

**Figure 4:** ROS content in myocardial cells detected using ELISA. (a) Micrograph. (b) Statistical diagram of ROS content. The ROS content in myocardial cells is markedly higher in the model group than that in the sham group, while it is markedly lower in the low-dose group and high-dose group than that in the model group. ^∗∗^*P* < 0.01 vs. model group, ^##^*P* < 0.01 vs. sham group.

**Figure 5:** Expressions of apoptosis-related proteins in myocardial cells determined using Western blotting. (a) Protein bands. (b) Expression level of Caspase-3. (c) Bcl-2/Bax. The model group has a remarkably increased expression of Caspase-3 and a remarkably decreased Bcl-2/Bax ratio compared with the sham group. Compared with the model group, the low-dose group and high-dose group have a remarkably decreased expression of Caspase-3 and a remarkably increased Bcl-2/Bax ratio. ^∗∗^*P* < 0.01 vs. model group, ^##^*P* < 0.01 vs. sham group.

**Figure 6:** Expressions of ERK pathway-related proteins in myocardial cells determined using Western blotting. (a) Protein bands. (b) Expression level of p-ERK. (c) Expression level of NF-*κ*B. The expression of p-ERK obviously declines and the expression of NF-*κ*B obviously rises in the model group compared with those in the sham group. The expression of p-ERK is significantly higher and the expression of NF-*κ*B is significantly lower in the low-dose group and high-dose group than those in the model group. ^∗∗^*P* < 0.01 vs. model group, ^##^*P* < 0.01 vs. sham group.

**Table 1:** Survival rate of rats at 7 d after MI.

Group	*n*	Survival rate
Sham group	10	100%
Model group	10	70%^#^
Low-dose group	10	90%^∗^
High-dose group	10	90%^∗^

Note: ^∗^*P* < 0.05 vs. model group, ^#^*P* < 0.05 vs. sham group.

## Data Availability

The datasets used and/or analyzed during the current study are available from the corresponding author on reasonable request.
